RETRACTED

# Data Mining Method of Intelligent Market Management Based on Collaborative Recommendation Algorithm

**DOI:** 10.1155/2022/8561567

**Published:** 2022-09-13

**Authors:** Ziling Wu, Shi Wang, Yuanhang Cai

**Affiliations:** ^1^School of Finance and Economics, Hainan Vocational University of Science and Technology, Haikou 571126, China; ^2^Public Teaching Department, Hainan Vocational University of Science and Technology, Haikou 571126, China; ^3^Chivast Education, Haikou Jiahua Education Consulting Co., Ltd., Haikou 570000, China

## Abstract

In order to solve the problems of low coverage and accuracy and large mean absolute error and root mean square error when traditional algorithms recommend market management data, this paper proposes an intelligent market management data mining method based on a collaborative recommendation algorithm. According to the preference value of the attribute characteristics of market management data, predict and score the attribute characteristics of market management data; use data mining technology to preprocess the information of market management data, combined with the design of collaborative filtering recommendation algorithm; and realize the collaborative filtering recommendation of market management data. With 50 recommendations, AGCAN improves the accuracy of MovieLens-1M by 43.81%, 5.43%, 1.87%, 0.42%, and 1.67%, respectively, compared with the five benchmark algorithms. For MovieLens-100K, compared with the five benchmark algorithms, AGCAN improves the accuracy by 51.17%, 10.52%, 3.37%, 0.1%, and 0.30%, respectively. Compared with the five benchmark algorithms, Amazon-baby and AGCAN have improved the accuracy by 34.37%, 28.12%, 31.25%, 29.1%, and 3.12%, respectively. The algorithm proposed in this paper uses a graph neural network to mine useful information between users and projects, but it lacks the use of other personalized interest information of users, such as user interest, user purchase time, and so on.

## 1. Introduction

With the continuous improvement of people's requirements for the quality of life, many network service platforms came into being. The service scale and the number of users provided by network platforms such as online film and sales are huge. There is a large amount of information related to films and commodities and the speed of information updates is fast. At the same time, the recommendation information processing system can be used for the government service system to help the market management work. The problem of information overload has become increasingly serious, and the recommendation information processing system can effectively help solve the corresponding problem of information overload. A good recommendation information processing system must be a personalized system that can improve both user satisfaction and merchant product profit margin [1, 2]. For Internet users, the recommendation system can help users collect and further retrieve effective information that meets the needs of users from the massive data on the Internet, so as to further provide users with more personalized services and improve users' product experience. For businesses, how to recommend appropriate products for different users is also of great significance and role in improving the purchase rate of users' recommended products and the profit margin of businesses. For market supervision and management, it can better understand the product layout of merchants and customer needs. The accuracy of recommendation has always been an important indicator in the application field of recommendation information processing systems, which can facilitate businesses to calculate and evaluate whether the products recommended for users can satisfy users. However, with the popularization and development of a personalized recommendation system, in addition to improving the accuracy, the reliability of recommendations is also gradually required. Nowadays, with the rapid development of the Internet, more auxiliary information can be obtained through different channels. Research shows that making rational use of these auxiliary information and giving appropriate examples to communicate with users not only can improve the accuracy and credibility of a personalized recommendation system but also can greatly improve the possibility of recommending users to choose appropriate personalized recommended products by themselves and convenient and comprehensive supervision of product quality [3–5].

RETRACTED

## 2. Related Works

In the environment of the rapid development of artificial intelligence and big data, the process of “looking for” information by users in the past has changed into the process of “looking for” users by information. Therefore, the application prospect of recommendation system is becoming more and more extensive. The quality of a recommendation system is closely related to the recommendation algorithm. At present, the mainstream recommendation algorithms are mainly divided into many kinds: content-based recommendation, hybrid recommendation, collaborative filtering recommendation, association rule-based recommendation, and neural network-based recommendation. Because each recommendation algorithm has its advantages and disadvantages, how to avoid its disadvantages and expand its advantages has become a research hotspot of scholars at home and abroad. Because of its good scalability and maturity, the collaborative filtering algorithm has become the first choice of recommendation system. Collaborative filtering is simply to use the preferences of a group with similar interests and common experiences to recommend information of interest to users [6].

Gohari and others extended the matrix decomposition algorithm and proposed the neural cooperative filtering model (NCF), which greatly improved the nonlinear modeling ability of the model [7]. Badis and others proposed a collaborative filtering algorithm based on optimized user similarity, adding an element to the traditional cosine similarity to calculate the level difference between users. It is used to calculate the score grade difference between different users of the project. His work is mainly to improve the formula for calculating user similarity, which is used to improve user similarity by adding the balance factor and weight [8]. Hsu and others proposed to use of the matrix decomposition method for collaborative filtering recommendations. Its main idea is to synthesize the single user characteristic matrix of different strategies into a group matrix. Strategy I is used to synthesizing the group matrix after the decomposition of the user scoring matrix. Strategy II is used to synthesize the group matrix before decomposing the user scoring matrix. Strategy III adds weight to user characteristics before user scoring and finally decomposes the group score [9]. Song and others proposed a matrix decomposition model to add group information features. The algorithm adds the group information to the joint information matrix, generates score prediction by adding matrix information features, and finally fuses the minimum pain strategy with the average value strategy to generate a satisfactory balance strategy for user score fusion [10]. Cui proposed a method to calculate the influence of members on each other based on similarity. The influence of members called leaders on other members is much greater than that of ordinary members. Therefore, the research attempts to calculate the influence of leaders on members and uses fuzzy clustering and similarity measurement to find similar interests for preference fusion [11]. Watada and others proposed the VAE model of extended polynomial possibility (multi-VAE) and compared and analyzed the likelihood function of the polynomial and collaborative filtering recommendation algorithm. The results show that the model is very effective for collaborative filtering of implicit feedback [12].

In this paper, an adaptive neural graph convolution attention collaborative filtering (ANGCACF) algorithm based on an adaptive graph convolution neural network is proposed. The graph convolution neural network is used to extract the characteristics of users and projects, adaptively adjust the aggregation coefficients of users and projects, increase the adaptive filling matrix, redistribute the weight coefficients of users and projects through the attention mechanism, and make top-N recommendation. The main contributions of this paper are as follows: an adaptive aggregation method is proposed to aggregate user and project characteristics. This method can adaptively adjust the aggregation coefficient. At the same time, experiments show that the aggregation coefficient of adaptive users and projects contributes the most to ANGCACF. An adaptive filling matrix is proposed to fill in the missing values of users and items, reduce sparsity, and use the attention mechanism to readjust the weights of users and items to achieve the optimal weight. The experimental results show that the recommendation accuracy of using the attention-based adaptive filling matrix is better than that of not using the attention-based adaptive filling matrix. Based on the public data sets of two different scenes of film and shopping, the proposed algorithm is compared with the four benchmark algorithms of pop, DMF, NNCF, and NGCF. The experimental results show that the algorithm proposed in this paper is reasonable and effective.

RETRACTED

## 3. Research Methods

### 3.1. The Significance of “Internet +” Consumer Market Management

If the “Internet +” is applied to the government service system, it is the “Internet + traditional government model” or the “traditional government model + Internet.” According to different situations, conditions, scenarios, and other external factors, the combination or priorities are different to a certain extent; through big data resources, modern communication technology, and network channels to make the Internet and traditional government mode scientific, reasonable, and effective fully integrated, improve the traditional government work processing mode, so as to optimize the office mode and functions, to create a new government model. In the traditional industrial and commercial administration registration, there are many problems such as multilevel examination and approval, strict examination, multidepartment registration, and imperfect exit mechanism. This mode directly leads to the complicated and long cycle of enterprise registration, affects the market access efficiency of investors, and also increases the operating cost of enterprises. If applied on the Internet and mobile terminal, you can directly in the “online” related application information, submit relevant application materials, query late license results, directly save the application steps to the examination and approval authority, also do not have to submit a lot of paper materials, save a lot of intermediate links, and improve the efficiency of the registration. Information resource sharing is realized through big data, information technology, and network channels. The relevant examination and approval departments directly transmit and receive information through the network platform, greatly reducing the time cost and resource cost of the applicant in the registration process, and improving the market access efficiency of consumers.

RETRACTED

To this end, consumer market management departments want to greatly improve economic development, stabilize market order, and improve service efficiency in the new era, You have to integrate into the new era, Constantly integrating the “Internet +” technology, follow the trend of the times. Make full use of its traditional advantages, and take innovation, upgrading, coordination, green and sharing the future as the development concept to form a brand-new consumer market management concept. We will actively guide and encourage market innovation, regulate market order in an orderly manner, and better safeguard consumers' rights and interests. Actively expand the density and depth of integration between the Internet and the consumer market, promote the upgrading of the management mode of the consumer market, improve the service, credit, integrity, and efficiency of the market management department, and comprehensively improve the market management efficiency through various measures. Therefore, the market management data mining based on the recommendation system can easily and comprehensively understand the product quality of merchants and improve the efficiency of market management and supervision.

### 3.2. ANGCACF Algorithm

#### 3.2.1. The Overall Framework of the Algorithm

ANGCACF algorithm is mainly composed of two parts: extracting feature vectors of users and items based on adaptive graph convolution attention neural network (AGCAN) [13–15]. AGCAN neural network combines the adaptive filling matrix graph convolution attention neural network (AFMGCAN) and the aggregation coefficient adaptive graph convolution neural network (AACGCN). AGCAN neural network includes one hot coding of user and item scores, adding the aggregation coefficient of the adaptive filling matrix, attention mechanism, and adaptive graph convolution neural network, so as to iterate the feature vectors of users and items [16]; The collaborative filtering recommendation algorithm framework based on matrix decomposition completes the prediction of recommendation algorithm and model optimization. The inner product *y*(*U*, *I*) of the user and project eigenvector is used as the user's interactive bias value for the project, and the target user is recommended and predicted according to this value.

RETRACTED

#### 3.2.2. Adaptive Graph Convolution Attention Neural Cooperative Model

Suppose that given user set *U*={*u*_1_, *u*_2_, *u*_3_,…, *u*_*n*_} and item set *I*={*i*_1_, *i*_2_, *i*_3_,…, *i*_*n*_}, *n* and *m* are the total number of users and items respectively. The interaction matrix between the user and the project is defined as *EεM*^*m*×*n*^, where *E*_*ij*_=1 indicates that the user *u*_*i*_ has interacted with the project *i*_*j*_. The user project interaction diagram is generated based on the interaction between user set *U* and project set. The schematic diagram of user project interaction is shown in Figure 1. Conduct one-hot coding on the interaction matrix *E* and embed the one-hot coding according to a certain dimension to generate *e*_*u*1_^0^ and *e*_*i*1_^0^, where *e*_*u*1_^0^ represents the initial user feature vector and *e*_*i*1_^0^ represents the initial project feature vector [17, 18].

#### 3.2.3. Adaptive Filled Matrix Convolution Attention Neural Network

After combining the user adaptive filling matrix with the user eigenvector [19, 20],

(1) $$\begin{array}{c} e_{u2}^{0}=e_{u1}^{0}+\Lambda \left(R_{u}\right), \end{array}$$

where *R*_*u*_ is a random vector with the same dimension as the user feature vector *e*_*u*1_^0^, Λ(•) is an adaptive calculation function, the adaptive filling matrix is trained through the machine learning binary adaptive mean aggregation layer (adaptive avgpool2d), and *e*_*u*2_^0^ is the user feature vector after the combination of the adaptive filling matrix and the user feature vector [21, 22].

The attention mechanism used in the ANGCACF algorithm is self-attention mechanism. The combined user feature vector and item feature vector are calculated as follows:

(2) $$\begin{array}{c} \partial_{u}=\text{Softmax}\left(e_{u2}^{0}\right), \end{array}$$

(3) $$\begin{array}{c} e_{u}^{0}=\partial_{u}\cdot e_{u2}^{0}. \end{array}$$

The user feature vector and item feature vector are obtained through (1)–(3). The fusion method of the feature vector embedding layer in AGCAN is as follows:

(4) $$\begin{array}{c} e_{u}^{0}=\text{Softmax}\left(e_{u1}^{0}+\Lambda \left(R_{u}\right)\right)*\left(e_{u1}^{0}+\Lambda \left(R_{u}\right)\right). \end{array}$$

The user feature vector is finally processed according to the following equation:

(5) $$\begin{array}{c} e_{u}^{l}=LR\left(W_{1}^{l}e_{u}^{l-1}+\sum_{i\in N_{u}}\frac{1}{\sqrt{\left|N_{u}\right|\left|N_{i}\right|}}\left(W_{1}^{l}e_{u}^{l-1}+W_{2}^{l}\left(e_{u}^{l-1}⊕e_{i}^{l-1}\right)\right)\right), \end{array}$$

where *LR*(•) is the LeakyRel activation function; *W*_1_^*l*^ and *W*_2_^*l*^ are the weight vectors corresponding to the user feature vector of the *l*-th iteration; *N*_*u*_ and *N*_*i*_ are the number of one-hop neighbors of user *u* and item *i*, respectively; *e*_*u*_^*l*−1^ is the user feature vector after iteration *l* − 1; *e*_*i*_^*l*−1^ is the user feature vector after iteration *l* − 1; and *e*_*i*_^*l*^ is the user feature vector after the *l*-th iteration [23].

RETRACTED

The steps of aggregating project eigenvectors and aggregating user eigenvectors are the same. The iterative rule in matrix form (formula (6)) is

(6) $$\begin{array}{c} E^{l}=\Theta \left(\left(\Omega +I\right)E^{l-1}W_{1}^{l}+\Omega E^{l-1}⊕E^{l-1}W_{2}^{l}\right), \end{array}$$

where *E*^*l*^ ∈ *M*^(*m*+*n*)×*d*^ is the characteristic matrix of users and projects obtained after one iteration; *d* is the embedded dimension; *E*^0^ is the initial representation of *E* , which is composed of *e*_*u*2_^0^ and *e*_*i*2_^0^ splicing; Θ(•) is the nonlinear transformation function [24]; *I* is the identity matrix of user and project interaction matrix; and Ω is the Laplace matrix of user and project interaction matrix. Its formula is as follows:

(7) $$\begin{array}{c} \Omega =D^{-0.5}AD^{-0.5}, \end{array}$$

where *A* is the adjacency matrix of the user and project interaction matrix and *D* is the degree matrix of user and project interaction matrix [25].

#### 3.2.4. Graph Convolution Neural Network with Adaptive Aggregation Coefficient

The user feature vector is processed according to the following equation:

(8) $$\begin{array}{c} e_{u}^{l}=LR\left(\left(1-\partial \right)W_{1}^{l}e_{u}^{l-1}+\partial \sum_{i\in N_{u}}\frac{1}{\sqrt{\left|N_{u}\right|\left|N_{i}\right|}}\left(W_{1}^{l}e_{u}^{l-1}+W_{2}^{l}\left(e_{u}^{l-1}⊕e_{i}^{l-1}\right)\right)\right), \end{array}$$

where *∂* is the adaptive adjustment aggregation coefficient calculated through the binary adaptive mean aggregation layer, and the binary adaptive mean aggregation layer does not share with the adaptive filling matrix, and the parameter is an independent calculation unit.

The steps of aggregating project eigenvectors and aggregating user eigenvectors are the same. The iterative rule in matrix form is as follows:

(9) $$\begin{array}{c} E^{l}=\Theta \left(\left(1-\partial \right)\left(\Omega +I\right)E^{l-1}W_{1}^{l}+\partial \Omega \;E^{l-1}⊕E^{l-1}W_{2}^{l}\right). \end{array}$$

#### 3.2.5. Adaptive Graph Convolution Attention Neural Network

Adaptive graph convolution attention neural network is composed of adaptive filling matrix graph convolution attention neural network and aggregation coefficient adaptive graph convolution neural network. As can be seen from Figure 2, AGCAN first obtains the relevant information about users and projects. By judging whether the sparsity of users and projects needs to enter the adaptive filling matrix convolution attention neural network when the sparsity is less than the adaptive threshold, AGCAN automatically enters the aggregation coefficient adaptive neural network to complete the aggregation of localized information. The processing flow of AGCAN feature vector aggregation is shown in Algorithm 1.

RETRACTED

### 3.3. Algorithm Prediction

User feature vector generated through 1-layer iteration. In {*e*_*u*_^0^, *e*_*u*_^1^, *e*_*u*_^2^,…, *e*_*u*_^*n*^}, the user feature vectors of different layers such as *e*_*u*_^0^ and *e*_*u*_^1^ reflect the different preferences and interests of users and connect the user feature vectors generated by all layers to generate the final feature vector of users. Similarly, the final feature vector of the project is also composed of the connection of the project feature vectors generated by multi-layer iteration. The eigenvectors of end users and projects are expressed as follows:

(10) $$\begin{array}{c} e_{u}^{*}=e_{u}^{0}\left\|\ldots \right\|e_{u}^{l},e_{i}^{*}=e_{i}^{0}\left\|\ldots \right\|e_{i}^{l}, \end{array}$$

where || represents the connection in the form of column as shown in the following formula:

(11) $$\begin{array}{c} e_{u}^{0}=\left[\begin{array}{cc} W & R\\ E & T \end{array}\right],\\ e_{u}^{1}=\left[\begin{array}{cc} S & F\\ D & G \end{array}\right],\\ e_{u}^{*}=e_{u}^{0}\|e_{u}^{1}=\left[\begin{array}{cc} W & RSF\\ E & T\;DG \end{array}\right]. \end{array}$$

Then, the final eigenvectors of the user and the project are processed by the inner product to obtain the user's preference $\bar{y}\left(U,I\right)$ for the project. The formula is defined as follows:

(12) $$\begin{array}{c} \bar{y}\left(U,I\right)=e_{u}^{*}\cdot e_{i}^{*}. \end{array}$$

### 3.4. Model Optimization

In order to optimize the parameters in the model, the loss function in the BPR recommendation algorithm is used to learn the parameters in the model. The BPR recommendation algorithm believes that the predicted value of positive sampling (users have historical interaction with the project) should be higher than that of negative sampling (users have no historical interaction with the project). The loss function of this model is as follows:

(13) $$\begin{array}{c} \text{Loss}=\sum_{\left(u,i,j\in \Omega \right)}-\ln\;\sigma \left({\bar{y}}_{ui}-{\bar{y}}_{uj}\right)+\tau {\left\|\theta \right\|}_{2}^{2}, \end{array}$$

where Ω={(*u*, *i*, *j*)*|*(*u*, *i*) ∈ Ω^+^, (*u*, *j*) ∈ Ω^−^} represents all data in the current data set, Ω^+^ is positive sampling sample data, Ω^−^ is negative sampling sample data, and *θ* is all trainable parameters in the model.

RETRACTED

At the same time, the Adam optimization algorithm is used to optimize the parameters in (13). Compared with the SGD optimization algorithm, the Adam optimization algorithm adds first- and second-order momentum, which is faster to find the local optimal solution.

### 3.5. Experimental Analysis

#### 3.5.1. Experimental Data Set

The experimental part uses real data sets from two different fields of film and shopping: MovieLens-1M, MovieLens-100K, and Amazon-book. Among them, MovieLens-1M and MovieLens-100K are collected by the GroupLens research team. MovieLens-1M is a benchmark data set for film recommendation scenes, which includes the explicit scores of about 100,000 users on the MovieLens website composed of 6,040 users and 3,952 films (the score range is 1∼5), and the sparsity is 95.81%. MovieLens-1M is a benchmark data set for film recommendation scenes. It includes about 1 million users on the MovieLens website, which is composed of 943 users and 1,682 movies. The score range is 1∼5, and the sparsity is 93.71%. Amazon-baby is a subset of the Amazon-review data set, including 531,890 users' 915,446 scores of 64,426 baby products, and the sparsity is 99.9973% (the score range is 1∼5).

The above two data sets are different in size and sparsity. In order to facilitate the experiment, the data sets are processed. First of all, the user will use the implicit feedback (which is greater than or equal to the value of 1) to show the positive feedback of the training items and use the implicit feedback (which is greater than or equal to the value of 1) to score the two items. Secondly, in MovieLens-1M, remove the project data with a score lower than 3, and the final data set contains 6,040 users, 3,629 movies, and 836,478 interactions. In Amazon-baby, because the data set is large and extremely sparse, and its quality is guaranteed by three core filtering, that is, users and projects with at least three interactions are retained. The final data set includes 52,672 users, 14,257 baby products, and 270,718 interactions. The statistics of MovieLens-1M and Amazon-book are shown in Table 1.

#### 3.5.2. Experimental Evaluation Index

In the experiment, the item set I generated by the recommendation algorithm is used for user *u*, where IU is for the *n*-th recommended item generated by user U. Define IR as the set of historical items that the user has actually selected in the test set and I as all test sets in the test set. The five indicators, Precision@N, Recall@N, NDCG@N, Hit@N, and Mrr@N, are used to evaluate the performance recommended by Top-N.

RETRACTED

A recall rate is a method to calculate the score of relevant items in all relevant items. The calculation formula is

(14) $$\begin{array}{c} \text{Recall}@N=\frac{I_{u}\cap I_{r}}{\left|I_{r}\right|}. \end{array}$$

The average reciprocal ranking is to calculate the ranking of the first relevant item found by the algorithm, which can be calculated by the following formula:

(15) $$\begin{array}{c} \text{Mrr}@N=\frac{1}{\left|I\right|}\sum_{u\in U}\frac{1}{{\text{rank}}_{u}^{*}}, \end{array}$$

where rank_*u*_^*∗*^ algorithm is the ranking position of the first relevant item found for the user.

The hit rate is a method to calculate how many hits there are in the *N*-size ranking item list. If at least one item is called a Hit in *I*, there is the following formula:

(16) $$\begin{array}{c} Hit@N=\frac{I_{u}}{I}. \end{array}$$

The purpose of the normalized impairment cumulative gain is to make the higher the ranking result, the more it can affect the final result. The calculation formula is as follows:

(17) $$\begin{array}{c} \text{NDCG}@N=\frac{\sum_{i=1}^{p}\left(2^{{\text{rel}}_{i}}-1/{\text{log}}_{2}i+1\right)}{\sum_{i=1}^{\left|\text{REL}\right|}\left(2^{{\text{rel}}_{i}}-1/{\text{log}}_{2}i+1\right)}, \end{array}$$

where rel_*i*_ represents the correlation degree at the position of *i* and |REL| means that the results are sorted in the order of relevance from large to small, and the set composed of the first *P* results is taken.

The accuracy rate can reflect the percentage of items of interest to users in the recommended items generated by the current recommendation algorithm. The calculation formula is as follows:

(18) $$\begin{array}{c} \text{Precision}@N=\frac{I_{u}\cap I_{r}}{\left|I\right|}. \end{array}$$

#### 3.5.3. Benchmark Algorithm and Experimental Setup

This experiment uses the following benchmark algorithms:

Pop (popularity) is recommended to users according to the popularity of items in the data set.

DMF is a deep structure learning architecture, which is based on the new loss function of cross entropy and fully considers the explicit rating and implicit feedback for a recommendation.

NNCF is a neural collaborative filtering model based on neighborhood, which integrates neighborhood information into the neural collaborative filtering method, including local information in user project interaction items, so as to make recommendations.

NAIS is a neural attention collaborative network, which uses the attention network to redistribute the weight coefficients in the historical interaction information between users and projects and then uses multi-layer perceptron to predict, so as to make recommendations.

RETRACTED

NGCF is a user item embedding neural network based on a depth map convolution neural network, which generates the characteristic information of users and items by multi-layer iteration of the localization information of users and items and then makes recommendations according to the collaborative filtering framework of matrix decomposition.

This paper completes the comparative experiment of AGCAN, AFMGCAN, AACGCN, and benchmark algorithm in the environment of Python3.8, PyTorch1.7.1, Cuda11.1.74, and RTX2060. In the experiment, according to the ratio of 8:1:1, the data set is randomly divided in the user dimension to construct the training set, verification set, and test set. The setting of superparameters of AGCAN, AFMGCAN, and AACGCN models is shown in Table 2. Set the default number of learning rounds (epochs) of the model to 300 and end the training in advance when the evaluation index on the verification set does not change within 10 rounds. The embedding dimension, learning rate, and batch size in the benchmark method are the same as AGCAN, AFMGCAN, and AACGCN, and other superparameters are consistent with the original paper or code by default. For the top-N recommendation task, set the number of recommendations *N* to {5,10,15,20,25,30,35,40,45,50}. The experimental goal is to recommend the top items for each user in the test set and use five indicators of Precision@N, Recall@N, NDCG@N, Hit@N, and Mrr@N to measure the performance of each model.

## 4. Result Analysis

### 4.1. Comparison with Benchmark Algorithm

Different top-N in the recommended task of the experiment will affect the test results. In order to carefully analyze and compare the index changes of AGCAN, AFMGCAN, AACGCN, and benchmark algorithm, the range of recommended quantity is set to 5∼50, and the interval is set to 5.

#### 4.1.1. Comparison of Recall and Accuracy

The experimental results of the algorithm and benchmark algorithm proposed in this paper on the Recall@N of MovieLens-1M, MovieLens-100K, and Amazon-baby data sets. The experimental results show that the Recall@N of AGCAN, AFMGCAN, AACGCN, and benchmark algorithm is directly proportional to the number of recommended items and tends to be flat with the increase of the number. The value of Precision@N tends to be inversely proportional to the number of recommended items. When the number of recommended items is 5, the recall rate gap between AGCAN, AFMGCAN, AACGCN, and benchmark algorithm is small, but with the increase in the number of recommended items, this gap gradually becomes larger. The recall rates of AFMGCAN and NGCF on MovieLens-1M are also relatively close, and the recall rates of AGCAN, AFMGCAN, AACGCN, and NGCF on MovieLens-100K are also relatively close. In Amazon-baby with extremely sparse data, the recommended recall rates of AGCAN, AFMGCAN, AACGCN, and NGCF have a large gap and are also higher than other benchmark algorithms. When the number of recommended items is 50, the accuracy gap between AGCAN, AFMGCAN, AACGCN, NAIS, and NGCF is small, but with the reduction of the number of recommended items, this gap gradually becomes larger. The accuracy of AFMGCAN and NGCF on MovieLens-1M is also close, and the accuracy of AGCAN, AFMGCAN, AACGCN, and NGCF on MovieLens-100K is also close. In Amazon-baby with extremely sparse data, there is a large gap in the recommended accuracy of AGCAN, AFMGCAN, AACGCN, and NGCF, which are also higher than other benchmark algorithms. The results show that AGCAN, AFMGCAN, and AACGCN perform well on data sets with large data sparsity.

RETRACTED

When the number of recommendations is 50, the recommendation performance of AGCAN, AFMGCAN, AACGCN, and benchmark algorithm is relatively good. Under this recommended number, for the experimental results of MovieLens-1M, compared with the five benchmark algorithms of pop, DMF, NNCF, NAIS, and NGCF, AGCAN has increased the value of Recall@50 by 47.95%, 3.70%, 2.45%, 2.02%, and 0.56%, respectively. For the experimental results of MovieLens-100K, compared with the five benchmark algorithms of pop, DMF, NNCF, NAIS, and NGCF, AGCAN has increased the value of Recall@50 by 56.04%, 9.34%, 3.22%, 1.56%, and 0.10%, respectively. For the experimental results of Amazon-baby, compared with pop, DMF, NNCF, NAIS, and NGCF, AGCAN has increased the value of Recall@50 by 27.28%, 24.26%, 28.46%, 37.52%, and 1.51%, respectively. A recall rate is a method to reflect the scores of items related to the recommendation algorithm. Therefore, with the increase of top-N, the recall rate also increases. The pop algorithm is only recommended to users according to popularity, without taking into account users' personalized interests, so its recall rate is the lowest: DMF, NNCF, NIAS, and NGCF algorithms take into account users' personalized interests and aggregate users' personalized interests through different methods, and their recall rate is higher than pop algorithm; AGCAN considers the problem of missing values of user and item eigenvectors and nonconvexity between the coefficients of aggregated users and items, so the recall rate of AGCAN is higher than that of pop, DMF, NNCF, and NGCF. Experimental data show that the recall rate of recommendation algorithm can be improved by further mining the potential information between users and projects.

RETRACTED

When the number of recommendations is 50, the recommendation performance of AGCAN, AFMGCAN, AACGCN, and benchmark algorithm is relatively good. Under this recommended number, for the experimental results of MovieLens-1M, compared with the five benchmark algorithms of pop, DMF, NNCF, NAIS, and NGCF, AGCAN has increased the value of Precision@50 by 43.81%, 5.43%, 1.87%, 0.42%, and 1.67%, respectively. For the experimental results of MovieLens-100K, compared with the five benchmark algorithms of pop, DMF, NNCF, NAIS, and NGCF, AGCAN has increased the value of Precision@50 by 51.17%, 10.52%, 3.37%, 0.1%, and 0.30%, respectively. For the experimental results of Amazon-baby, compared with the five benchmark algorithms of pop, DMF, NNCF, NAIS, and NGCF, AGCAN has increased the value of Precision@50 by 34.37%, 28.12%, 31.25%, 29.1%, and 3.12%, respectively. The accuracy rate reflects the percentage of items of interest to users in the recommended items generated by the current recommendation algorithm. Therefore, with the increase of top-N, the accuracy rate also decreases. Pop only considers the popularity of items and does not consider users' personalized interests, so pop has the lowest accuracy; DMF and NNCF both consider the cross information of users and projects, so the accuracy is higher than pop, and the accuracy value is not much different; NAIS and NGCF consider the aggregation of localized information and weight distribution among user items, so their accuracy is higher than pop, DMF, and NNCF; AGCAN solves coefficient resetting and localized information aggregation, so its accuracy is higher than all baseline algorithms. The experimental data show that the accuracy of the recommendation algorithm can be improved by further mining the potential information between users and projects.

#### 4.1.2. Comparison of Hit, NDCG, and MRR

According to the experimental results of recall and accuracy, the three recommendation algorithms proposed in this paper are close to the recommendation index of NGCF, and the recommendation index of NGCF is higher than other benchmark algorithms. Therefore, according to the experimental data, the improvement percentage of the model relative to NGCF when the number of recommendations is 50 is obtained, as shown in Table 3.

According to the data in Table 3, the recommended performance of the three algorithms is better than that of the baseline algorithm at the top-50, and the recommended performance of the three algorithms on the Amazon-baby data set is improved more, which proves that the three algorithms can alleviate the data sparsity to a certain extent.

#### 4.1.3. Algorithm Contribution

According to the data of MRR@50 and NDCG@50 in the experimental results, the contribution of AFMGCAN and AACGCN to AGCAN can be obtained. The analysis of model contribution is shown in Table 4.

RETRACTED

Table 4 calculates the performance contribution value of AFMGCAN and AACGCN to AGCAN according to formula (19). The closer the value obtained from this formula is to 0, the greater its contribution value to AGCAN. Through this formula, it is concluded that the contribution value of AACGCN to AGCAN is the largest in the data set with small sparsity, while the contribution value of AFMGCAN is larger in the data set with large sparsity. According to the above analysis of Precision@N, Recall@N, NDCG@N, Hit@N, and MRR@N, NGCF is localized information aggregation, NAIS is an attention neural network, and the performance of NGCF is higher than NAIS. AFMGCAN only considers the redetermination of parameter weights of missing data values and missing data values, while AFMGCAN considers the aggregation of localized information. Therefore, AACGCN contributes the most to the performance of AGCAN in the data set with large sparsity, while AFMGCAN contributes the most to the performance of AGCAN in the data set with small sparsity.

(19) $$\begin{array}{c} \text{RelativeOfImprove}=\frac{\text{Basic}-\text{Improve}}{\text{Basic}}. \end{array}$$

Through the comprehensive analysis of Tables 3 and 4, it can be concluded that:

- AGCAN, AFMGCAN, and AACGCN perform well in data sets with large sparsity and are much higher than other benchmark algorithms. Experiments show that the three algorithms proposed in this paper can solve the sparsity problem to a certain extent.
- Sparsity has a great impact on the performance of the recommendation algorithm. The sparsity of the Amazon-baby data set is the largest, resulting in the performance of all recommendations being inferior to MovieLens-100K and MovieLens-1M data sets.
- AACGCN contributes the most to the performance of AGCAN in the data set with large sparsity, while AFMGCAN contributes the most to the performance of AGCAN in the data set with small sparsity.
- The performances of AGCAN, AFMGCAN, and AACGCN are better than NGCF. At the same time, the three algorithms proposed in this paper are variants of NGCF.

### 4.2. Influence of Localization Information Aggregation Order

In order to study the influence of localization information aggregation order on recommendation performance, set localization information aggregation order *l* to {1,2,3,4} and conduct experiments on MovieLens-100K, MovieLens-1M, and Amazon-baby data sets. At the same time, Hit@10 and Precision@10 are used to evaluate the impact of different orders of models, and other parameters remain unchanged by default.

RETRACTED

As shown in Table 5, under the condition of top-10, with the increase of embedding and localization information aggregation order *L*, the hit rate and accuracy of the three data sets are improved to a certain extent. In Amazon-book, the improvement percentage of the two indicators is significantly higher than MovieLens-1M. This is because when the interactive data is very sparse, increasing the aggregation order of localized information can enable the model to mine deeper information, so as to enrich the internal characteristics of the project and reduce the negative impact of sparsity on recommendation performance.

### 4.3. Influence of Negative Sampling Rate on the Model

Negative sampling will update a small part of the weight of the model to optimize the recommendation performance of the model. In order to analyze the influence of the number of negative samples on the experimental results, the range of negative sampling rate is set to {1,3,5,7,9}. Experiments were carried out on MovieLens-100K, MovieLens-1M, and Amazon-baby data sets, and models with different negative sampling rates were evaluated by using Hit@10 value and NDCG@10. Experiments were carried out on MovieLens-100K, MovieLens-1M, and Amazon-baby data sets, and other parameters remained unchanged by default. The experimental results of Hit@10 and NDCG@10 values of AGCAN, AFMGCAN, and AACGCN models under different negative sampling rates are shown in Figures 3(a)–3(c) and 4(a)–4(c). When the number of negative samples is set to 1, AGCAN, AFMGCAN, and AACGCN models have performed well on MovieLens-100K and Amazon-baby data sets. However, on the MovieLens-100K data set, the recommended performance is not affected by negative sampling, because the sparsity of the MovieLens-100K data set is not as large as that of the MovieLens-1M and Amazon-baby data sets, and the data volume is not as large as that of the MovieLens-1M and Amazon-baby data sets, so a small number of negative samples cannot have sufficient impact on the model. With the increase of the number of negative samples, the performance of the model will become better to a certain extent. However, the experimental results show that increasing too many negative samples will lead to performance degradation. When the number of negative samples is 1 or 3, the values of Hit@10 and NDCG@10 on MovieLens-1M and Amazon-baby data sets are relatively the highest. When the negative sampling rate is 1, the value of Hit@10 is the best, and then the performance begins to decline. When the negative sampling rate is 3, the value of NDCG@10 is the best, and then the performance begins to decline. Note that the performance of the model also shows the same change trend as MovieLens-1M on Amazon-book. Using a certain negative sampling strategy can balance the proportion of positive and negative samples, so as to update the weight of a part of the model to optimize the recommendation performance of the model and improve the recommendation performance. However, too many negative samples will deteriorate the robustness of the model and reduce the recommendation performance; it is difficult to obtain the optimal results and waste a lot of time reading negative samples. Therefore, the best range of negative sampling rate of the model is {1,3}.

RETRACTED

## 5. Conclusion

This paper proposes an adaptive graph convolution attention neural collaborative recommendation algorithm, which is applied to market management data mining. The graph neural network is combined with the collaborative filtering framework. The improved collaborative recommendation algorithm is used to extract the feature information from the local information of users and projects and jointly learn the user and project representation in the end-to-end model, which effectively alleviates the problem of sparsity and improves the accuracy of recommendation. Experiments are carried out on three real movie and shopping data sets, Movielens-1M, Movielens-100K, and Amazon-book. Precision, recall, MRR, hit, and NDCG are used as the evaluation indexes of the model, and the algorithm proposed in this paper is compared with pop, DMF, NNCF, NAIS, and NGCF. The experiments show that the indexes of the algorithm proposed in this paper are better than the comparison algorithm on the three data sets and can provide users and market management agencies with more accurate recommendation results.

## Figures and Tables

**Figure 1:** User project interaction diagram.

**Figure 2:** AGCAN algorithm flow.

**Figure 3:** Hit rate under negative sampling.

**Figure 4:** NDCG under negative sampling.

**Algorithm 1:** AGCAN algorithm.

**Table 1:** Statistics of experimental data set.

Data set		MovieLens-1M	Amazon-baby	MovieLens-100K
User project interaction	#ofuses	6,040	52,672	943
	#ofitems	3,629	14,257	1,682
	#ofinteractions	836,478	270,718	100,000
	#sparsity (%)	96.10	99.96	93.71

**Table 2:** Superparameter setting of the model.

Superparameter name	Parameter value
User and item embedding dimension	64
Optimizer	Adam
Learning rate	0.001
Batch size (trainbatchsize)	2,048
L2 regular term coefficient	1*e* − 2
Weight_decay	0.0

**Table 3:** Percentage increase of model top-50 relative to NGCF.

Model		AGCAN	AFMGCAN	AACGCN
MovieLens-100K	Recall	0.11	0.82	0.32
	MRR	1.41	2.04	1.74
	NDCG	3.02	1.95	1.63
	Hit	0.38	0.38	0.38
	Precision	0.3	1.844	1.02

MovieLens-1M	Recall	0.57	0.55	2.02
	MRR	0.5	0.09	0.4
	NDCG	0.24	0.07	0.76
	Hit	0.33	0.15	1.02
	Precision	0.64	1.06	0.53

Amazon-baby	Recall	6.78	2.4	6.7
	MRR	12.39	9.29	8.85
	NDCG	14.21	4.98	7.73
	Hit	5.479	3.22	6.64
	Precision	6.58	3.22	6.45

RETRACTED

**Table 4:** Model contribution analysis.

Model		AGCAN	AFMGCAN		AACGCN	
MovieLens-100K	MRR@50	**0.4193 (1.41%)**	0.4192	(0.49%)	0.4209	(0.09%)
	NDCG@50	**0.2916 (3.02%)**	0.2911	(0.17%)	0.2931	(−0.51%)

MovieLens-1M	MRR@50	**0.5026 (0.5%)**	0.5017	(0.17%)	0.5022	(0.07%)
	NDCG@50	**0.3846 (0.24%)**	0.3806	(1.04%)	0.3794	(1.35%)

Amazon-baby	MRR@50	**0.0254 (12.39%)**	0.0247	(2.75%)	0.0246	(3.14%)
	NDCG@50	**0.0458 (14.21%)**	0.0421	(8.07%)	0.0432	(5.67%)

**Table 5:** Effect of aggregation order of localized information on recommendation performance.

Algorithm	AGCAN		AFMGCAN		AACGCN	
	Hit@10	Precision@10	Hit@10	Precision@10	Hit@10	Precision@10
MovieLens-100K	0.7091	0.1708	0.7119	0.1713	0.7126	0.1723
	0.7142	0.1731	0.7154	0.174	0.7167	0.1748
	0.7109	0.1742	0.7195	0.1752	0.72	0.1756
	0.7122	0.1762	0.7152	0.1754	0.7221	0.1776

MovieLens-1M	0.0463	0.0045	0.0465	0.0048	0.0475	0.0049
	0.0479	0.0049	0.0536	0.0055	0.0529	0.0055
	0.051	0.0052	0.0574	0.0059	0.0585	0.0059
	0.0525	0.0055	0.0576	0.0061	0.0609	0.0059

Amazon-baby	0.7818	0.199	0.7828	0.1999	0.7736	0.1934
	0.7836	0.1996	0.7885	0.2021	0.7785	0.1994
	0.7852	0.2007	0.7985	0.2025	0.7805	0.2009
	0.7985	0.2023	0.8028	0.207	0.7911	0.2017

## Data Availability

The data sets used and/or analyzed during the current study are available from the corresponding author on reasonable request.
